# Abnormal Variations of the Key Genes in Osteoporotic Fractures

**DOI:** 10.1155/2022/1022078

**Published:** 2022-10-29

**Authors:** Bin Wang, Caiyuan Mai, Lei Pan

**Affiliations:** ^1^Department of Orthopedics, Foshan Sanshui District People's Hospital, Foshan 528100, China; ^2^Department of Obstetrics, Guangdong Women and Children's Hospital, Guangzhou 510010, China

## Abstract

**Objective:**

The classical osteoporotic signaling pathways include the four key genes (LRP5, Runx2, Osterix, and RANKL) influencing the regulation of osteogenesis and osteoclastogenesis. This study investigates the expression of these four genes associated with bone remodeling during fracture healing.

**Methods:**

Ovariectomized rats as an osteoporotic group were randomly divided into three groups-group A, group B, and group C. Nonosteoporotic rats as the control group were likewise divided into three groups A0, B0, and C0, using the same method. The rats were killed on the third day of fractures in groups A and A0, on the seventh day of fractures in groups B and B0, and on the fourteenth day of fractures in groups C and C0. The bone specimens were taken from the femoral fracture site, and the expression level of each gene in the bone specimens was detected using RT-qPCR, Western blotting, and immunohistochemistry.

**Results:**

LRP5, Runx2, and Osterix expressions were decreased in osteoporotic rat fractures and then increased over time. The expression of RANKL was elevated in osteoporotic rat bone specimens, which decreased after that.

**Conclusion:**

The expressions of the four genes varied with time after fracture, which could be associated with the various stages of bone repair. The four genes can inform practice in ideal interventions in the prevention and management of osteoporosis.

## 1. Introduction

Osteoporosis is a metabolic disorder associated with systemic bone aging and degradation. Osteoporosis is characterized by decreased bone mass, structural degradation, increased brittleness, and susceptibility to fractures [1]. Worldwide, one in five men over the age of 50 years sustained an osteoporotic fracture (OPF) in 2020 [2]. Fracture is the most serious outcome of osteoporosis. Postmenopausal osteoporosis (PMOP) occurs in women after menopause due to estrogen deficiency, resulting in bone loss and bone structure changes. Osteoporosis is three times more common in postmenopausal women than in non-postmenopausal women [3]. PMOP can significantly increase disability rates and mortality rates and result in a great family and socioeconomic burdens [4, 5]. The process of osteoporotic development involves bone resorption mediated by osteoclast and bone formation mediated by osteoblast, which maintains the bone in a state of continuous remodeling. Under physiological conditions, bone absorption and formation remain stable; however, osteoporosis develops when the balance is disrupted, where the bone resorption rate is higher than the formation rate [6, 7].

Osteogenesis and osteoclastogenesis have been the subjects of interest in osteoporosis. The classical Wnt/*β*-catenin, BMP-2/Osterix, and RANKL/RANK signaling pathways include the key genes influencing the regulation of osteogenesis and osteoclastogenesis. LRP5, Runx2, and Osterix are the key osteogenic genes associated with the Wnt/*β*-catenin and BMP-2/Osterix signaling pathway, while RANKL is a key gene associated with the RANKL/RANK signaling pathways [8, 9]. However, the evolving process of these genes in osteoporotic fracture remains unclear. Therefore, the overall aim of the present study was to investigate the genes associated with the development and healing stages of osteoporotic fractures based on histological and molecular analyses of fracture healing stages. Specifically, this study aimed to investigate the variations of LRP5, Runx2, Osterix, and RANKL in bone specimens using RT-qPCR and immunohistochemistry.

## 2. Materials and Methods

Following the Animal Experimentation Ethics Guidelines, the Ethics Committee of Foshan Sanshui District People's Hospital approved the procedures of the study (Medical Research in Guangdong Province 2019003). A total of 100 Sprague–Dawley female rats (12 weeks old, weighing 200–220 g) were purchased from the Guangzhou medical university. Then, the rats were housed in a specific pathogen-free (SPF) facility (temperature 22 ± 2°C; humidity 50 ± 10%) with a 12/12-h light/dark cycle, and standard laboratory animal food and tap water were available ad libitum. First, the rat model of an osteoporotic model of ovariectomy (OVX)-induced osteoporosis was established by removing the ovaries bilaterally, and then, after 12 weeks, we selected 90 rats weighing 280–300 g. Another 90 rats of the same age and weight were purchased as a control group (without being subjected to sham procedures). A micro-CT (Perkin Elmer, China) for small animals was used to determine the femur bone mineral density (BMD) in all rats. Ovariectomized rats were sure to be Osteoporotic rats. With the anesthetic, an osteotomy was established using an oscillating sagittal saw at the left proximal femur in all rats, and then the incision was closed. Ninety osteoporotic rats were randomly divided into groups A, B, and C, with 30 cases in each group. Ninety nonosteoporotic rats were randomly divided into groups A0, B0, and C0, with 30 cases in each group. The rats were killed on the third day of fractures in groups A and A0, on the seventh day of fractures in groups B and B0, and on the fourteenth day of fractures in groups C and C0. A bone specimen was taken from the fractured femur when the rats were killed. Specimens (the bone tissues were equal to or more than 400 mg and the intercepted bone mass was greater than 0.8 cm × 0.3 cm × 0.3 cm in volume) were collected from the fracture sites. Specimens were collected and stored immediately in liquid nitrogen.

### 2.1. RT-qPCR

Briefly, 100 mg of bone tissue was first ground in liquid nitrogen. Total RNA was then extracted from the bone tissues using the RNAiso Plus kit (Duoyang, China). cDNA was synthesized from the RNA using PrimeScript RT Master Mix (TaKaRa, Japen). The DNA was amplified using Real-time PCR (RT-qPCR) with the SYBR Premix kit (TaKaRa, Japen). Primers used in this research were synthesized by Thermo Fisher Scientific company. Conditions of PCR were as follows: initial denaturation at 94°C for 5 minutes, 30 elongation cycles at 94°C for 30 seconds, annealing at 58°C for 30 seconds, extension at 72°C for 40 seconds, and final extension at 72°C for 10 minutes. GAPDH was used as the internal control. The amplification of the DNA was expressed based on the Ct (2^−ΔΔCT^) equation.

### 2.2. Western Blotting (WB)

Same with the aforementioned method, 200 mg of bone tissue was ground. Total protein was extracted from bone tissues using RIPA lysis buffer (Beyotime, China). The protein concentration was determined using a BCA assay kit (Beyotime, China). A total of 30 *µ*g protein/well was resolved using 10% SDS-PAGE and transferred to a PVDF membrane. Subsequently, 5% nonfat milk was used to block the membrane at 37°C for 1 h, followed by incubation at room temperature for 1 h with primary antibodies (Abcam, UK., LRP5 antibody: no. ab223203; Runx2 antibody: no. ab92336; Ostrix antibody: no. ab209484; RANKL antibody: no. ab239607; GAPDH antibody: ab8245). The membrane was then incubated with horseradish peroxidase-conjugated anti-rabbit IgG secondary antibody (Abcam, UK., ab150113) at room temperature for 2 h. The bands were visualized by using enhanced chemiluminescence (ECL) reagent kit (Yeasen, China) and semiquantified with Image J software.

### 2.3. Immunohistochemical Analysis

Intercepted bone mass was thawed, fixed in 10% neutral formalin for 48 hours, and embedded in paraffin after decalcification in 10% EDTA solution (Zhongshan Jinqiao, China). The specimens were then cut into 5 *μ*m thick sections and treated with 3% hydrogen peroxide for 10 min. Afterward, the sections were rinsed with phosphate-buffered saline, incubated with primary and secondary antibodies (Abcam, UK., the same as WB) sequentially, and exposed to DAB (TaKaRa, Japen). The sections were counterstained with hematoxylin solution (TaKaRa, Japen). Ten visual fields were randomly selected and observed under a high magnification microscope (Olympus, Japen), and the number of positively stained cells was calculated.

### 2.4. Data Analysis

All experiments were performed at least three times. Continuous data were expressed as mean ± standard deviation (±*s*). A one-way analysis of variance was used for multigroup comparison, and differences between the two groups were determined by LSD *t*-test. *P* < 0.05 was considered statistically significant. Data were analyzed using GraphPad Prisma 5 software and SPSS V. 22.0 (Chicago, USA).

## 3. Results

### 3.1. Weight and BMD of Rats

None of the rats died during the experiment. The weights (g) of groups A, B, C, A0, B0, and C0 were: 285.3 ± 2.5, 287.3 ± 3.6, 283.6 ± 7.4, 284.6 ± 6.2, 287.3 ± 8.9, and 286.5 ± 8.0, respectively, and no significant differences existed between any two groups (*P* > 0.05). The weights (g) of the whole osteoporotic and control groups were 286.3 ± 6.4 and 286.0 ± 2.6, without significant differences (*P* > 0.05).

The values of BMD (g/cm^2^) of groups A, B, C, A0, B0, and C0 were 0.42 ± 0.25, 0.44 ± 0.06, 0.43 ± 0.14, 0.21 ± 0.02, 0.23 ± 0.09, and 0.22 ± 0.08, respectively. There were no significant differences between any two groups in groups A, B, and C, and there were no significant differences between any two groups in groups A0, B0, and C0 (*P* > 0.05). The values of BMD (g/cm^2^) of the whole osteoporotic group and control group were 0.43 ± 0.18 and 0.22 ± 0.05, and there was a significant difference between them (*P* > 0.05).

### 3.2. Expressions of LRP5, Runx2, Osterix, and RANKL in the Groups (Osteoporotic Group and Control Group) Using RT-qPCR

RT-qPCR results revealed that the levels of LRP5, Runx2, and Osterix in the bone tissues were lower in the osteoporotic group than in the control group (*P* < 0.05), while the level of RANKL was higher in the osteoporotic group than in the control group (*P* < 0.05) (Figure 1).

### 3.3. Expressions of LRP5, Runx2, Osterix, and RANKL in the Groups Using RT-qPCR and WB

The levels of LRP5, Runx2, Osterix, and RANKL between groups A0 and A, B0 and B, and C0 and C exhibited a highly significant difference (*P* < 0.05). However, the differences between groups A0, B0, and C0 were insignificant across the four genes (*P* > 0.05). The elevated expressions of LRP5 and Runx2 were found lowest in group A (the third day) than in groups B (the seventh day) and C (*P* < 0.05), and the elevated expressions of Osterix were highest in group C (the fourteenth day) than in groups A and B (*P* < 0.05), while the depressed expressions of RANKL were highest in group A (the third day) than in groups B and C (*P* < 0.05). The differences in LRP5 and Runx2 between groups B and C, Osterix between groups A and B, and RANKL between groups B and C were not found to be significant (*P* > 0.05) (Figures 2–4).

### 3.4. Immunohistochemical Staining of Proteins in LRP5, Runx2, Osterix, and RANKL

The image of immunohistochemical staining is visible in Figures 5 and 6. The number of positively stained cells was calculated. The levels of LRP5, Runx2, Osterix, and RANKL are the same variations as the above.

## 4. Discussion

Patients with osteoporosis are prone to occur OPF [10]. There was a 20 percent chance of death with complications of osteoporosis, and 20 percent or so of patients with recurrent fractures in the proximal femur of OPF [11]. In China, ∼83.9 million people are estimated to suffer from osteoporosis, and this number, including osteopenia, should increase to ∼212 million people by 2050 [12]. Osteoporosis and postmenopausal osteoporotic fracture (PMOPF) have globally become critical public health problems. The present study investigated the relationships of mRNA and protein expressions in LRP5, Runx2, Osterix, and RANKL in bone specimens of osteoporotic rats.

Osteogenesis and osteoclastogenesis are regulated by the Wnt/*β*-catenin, BMP-2/Runx2/Osterix, and RANKL/RANK signaling pathways [8, 9, 13–17]. Based on histological and molecular analyses, the early stage of fracture healing can be divided into the early inflammatory response stage (one day after fracture), the nonspecific bone anabolic stage (three days after fracture), the nonspecific catabolic stage (three days to one week after fracture), and the specific bone anabolic stage (more than one week after fracture). The entire fracture healing phase can be divided into three stages: hematoma organization, original callus formation, and callus reconstruction molding stage. The hematoma organization stage is typically completed within 2 weeks after fracture [18, 19]. Consequently, we stratified osteoporotic rats into several groups to reflect the healing stages Group A (the third day), B (the seventh day), and C (the fourteenth day). The control group was divided into A0 to C0 using the method noted above. Our results depicted that LRP5, Runx2, and Osterix expressions decreased in osteoporotic rat fractures and then increased with the increase over time. The expression of RANKL was elevated in osteoporotic rat bone specimens, which decreased after that.

In the Wnt/*β*-catenin signaling pathway, the Wnt, LRP5/6, and FZD complexes recruit Dvl and degradative complexes, which inhibit the phosphorylation of *β*-catenin by GSK-3*β*. Accumulating nonphosphorylated *β*-catenin in the nucleus activates downstream Runx2 and other genes, resulting in osteogenesis [8, 20]. LRP5 exists on the surface membranes of numerous cells [21]. Inhibition of LRP5 impairs the proliferation of osteoblasts, affecting bone formation [22]. Glinka [23] revealed that LGR5 regulated embryonic patterns and the proliferation of stem cells through the Wnt/*β*-catenin mediated agonist of *R*-cavernous signaling. In the present study, we observed substantial underexpression of LRP5 in the bone specimens of osteoporotic rats, which was consistent with the above theory. Runx2 is a highly specific biomarker for osteogenesis. The expression of Runx2 is essential for bone formation and development. In particular, Runx2 upregulates the transcription of genes for several mineralization-related genes in osteoblasts [24, 25]. The Wnt/*β*-catenin pathway directly regulates Runx2, strengthens osteogenic differentiation, and accelerates fracture healing [24]. In the present study, we observed a significant underexpression of Runx2 in osteoporotic rats, which reflects inadequate osteogenesis in osteoporotic rats.

LRP5 regulates osteoblastosis and bone formation by activating the expression of Runx2 [26]. The expression levels of LRP5 and Runx2 were simultaneously lowest in group A and then went up synchronously in groups B and C, which suggests that variations of LRP5 and Runx2 were consonantly correlated with the given osteogenic stage.

BMP-2 modulates the transcription of the BMP-2/Runx2/Osterix pathway by activating the expression of Smads [27]. Smads regulate the transcription of several target genes and induces the expression of Runx2. Osterix is a key osteogenic gene downstream of Runx2 [28], and Runx2 can upregulate the expression of Osterix [29]. Osterix was underexpressed in osteoporotic rats, suggesting that it is a critical downstream osteogenic gene that influences the healing of osteoporotic fractures.

A study that used mouse models revealed that cartilage and bone specimen formation commences seven days after fracture and is sustained until the tenth day [30]. Osterix was generally expressed in the osteoblasts adjacent to the injury site fourteen days after fracture, which promoted the hardening of cartilage at the injured site; furthermore, numerous studies have demonstrated that BMP exerts a unique osteogenic effect, which fixes the fiber junction within two weeks after fracture [8, 9]. In the present study, the elevated expressions of Osterix were highest in group C (the fourteenth day) than in groups A and B, which was consistent with the findings.

The OPG/RANKL/RANK pathway is essential for regulating the differentiation of osteoclasts, including the expressions of RANKL, RANK (on the respective cell membranes), and OPG (a pseudoreceptor). Given the high affinity between OPG and RANKL, OPG can competitively inhibit the interaction of RANKL and RANK, further disrupting the differentiation of osteoclasts [10]. The differentiation and maturation of osteoclasts are exclusively stimulated by RANKL [31]. We observed that RANKL was overexpressed in osteoporotic fractures, consistent with previous findings [32]. Expressions of RANKL were highest in group A (the third day after fracture), which decreased after that, reflecting the role of RANKL in osteoclasts and the healing process of osteoporotic fractures.

Although we did not investigate the mechanisms underlying the abnormal variations of LRP5, Runx2, Osterix, and RANKL in the bone specimens of osteoporotic rats, our findings provided strong evidence that the Wnt/*β*-catenin, BMP-2/Runx2/Osterix, and RANKL/RANK pathways regulated osteogenesis and osteoclastogenesis in osteoporotic fractures of rats. The expressions of the four genes associated with bone remodeling during fracture healing varied with time after fracture, which could be associated with the various stages of bone repair. The characteristic variations in the expression of the four genes may inform future ideal interventions in preventing PMOP and managing PMOPF.

## Figures and Tables

**Figure 1:** Relative expressions value of mRNA of LRP5, Runx2, Osterix, and RANKL in bone tissues of control and osteoporotic groups. ^#^*P* < 0.05.

**Figure 2:** Relative expressions value of mRNA of LRP5, Runx2, Osterix, and RANKL in bone tissues of groups A0, B0, C0, A, B, and C ^#^*P* < 0.05.

**Figure 3:** Western blotting was performed to determine protein expressions of LRP5, Runx2, Osterix, and RANKL in bone tissues of groups A0, B0, C0, A, B, and C ^#^*P* < 0.05.

**Figure 4:** Relative protein expressions value of LRP5, Runx2, osterix, and RANKL in bone tissues of groups A0, B0, C0, A, B, and C ^#^*P* < 0.05.

**Figure 5:** Immunohistochemical staining of LRP5, Runx2, Osterix, and RANKL in bone mass of participants in groups A0, B0, C0, A, B, and C. The legend of scale bar = 50 *μ*m.

**Figure 6:** A histogram representing quantitative analysis results of immunohistochemical staining in LRP5, Runx2, Osterix, and RANKL in bone specimens (groups A0, B0, C0, A, B, and C. ^#^*P* < 0.05.

## Data Availability

The datasets used or analyzed during the current study can be obtained from the corresponding author upon reasonable request.

## Abbreviations

PMOPF: Postmenopausal osteoporotic fracture
PMOP: Postmenopausal osteoporosis
OPF: Osteoporotic fracture.
